# Design and Simulation Analysis of a Robot-Assisted Gait Trainer with the PBWS System

**DOI:** 10.1155/2021/2750936

**Published:** 2021-11-15

**Authors:** Jiancheng (Charles) Ji, Yufeng Wang, Guoqing Zhang, Yuanyuan Lin, Guoxiang Wang

**Affiliations:** ^1^Institute of Intelligent Manufacturing, Shenzhen Polytechnic, 4089 Shahe West Road, Shenzhen 518055, China; ^2^People's Hospital of Gaoxin, 768 Fudong Road, Weifang 261205, China; ^3^Weifang Hospital of Traditional Chinese Medicine, 1055 Weizhou Road, Weifang 261042, China; ^4^Soochow University, 50 Donghuan Road, Suzhou 215301, China

## Abstract

In response to the ever-increasing demand of lower limb rehabilitation, this paper presents a novel robot-assisted gait trainer (RGT) to assist the elderly and the pediatric patients with neurological impairments in the lower limb rehabilitation training (LLRT). The RGT provides three active degrees of freedom (DoF) to both legs that are used to implement the gait cycle in such a way that the natural gait is not significantly affected. The robot consists of (i) the partial body weight support (PBWS) system to assist patients in sit-to-stand transfer via the precision linear rail system and (ii) the bipedal end-effector (BE) to control the motions of lower limbs via two mechanical arms. The robot stands out for multiple modes of training and optimized functional design to improve the quality of life for those patients. To analyze the performance of the RGT, the kinematic and static models are established in this paper. After that, the reachable workspace and motion trajectory are analyzed to cover the motion requirements and implement natural gait cycle. The preliminary results demonstrate the usability of the robot.

## 1. Introduction

Along with development of the aging society, the lower limb rehabilitation demands of the elderly and the pediatric patients with neurological impairments are getting larger [1] and there are at least 36 million disabilities reported by the World Health Organization in 2016 [2]. For pediatric patients suffering from stroke, traumatic brain and spinal cord injuries, infantile cerebral palsy, and Parkinson's disease, mobility and balance are the essential factors in the Activities of Daily Living (ADL) [3]. But, those patients usually suffering from dyskinesia and balance function disorder require systematic rehabilitation treatments, such as gait training and balance training, to perform specific movements [4]. Large-scale rehabilitation equipment is advantageous in the earlier intervention treatments via continuous passive motion training, which is beneficial to prevent adhesion and stiffness of joints and recover function of joint movement after arthrolysis [5]. However, previous experience revealed that the traditional robots face problems due to the suspension BWS and lower extremity exoskeleton, such as the limitation of pelvic motions which affects the natural gait [6].

To date, different types of lower limb rehabilitation robots have been developed to improve mobility and balance function by the intervention of robotic technology [7–10]. The lower limb rehabilitative robots are mainly divided into two major categories: (i) mobile type and (ii) stationary type. The mobile type contains joint level device, portable exoskeleton, the BWS with mobile base, and so on. The stationary type contains body weight support (BWS) with a treadmill, the BWS with an exoskeleton, the BWS with a footplate device, and so on. For the shortage in active control of the lower limbs, mobile walkers are not suitable for early treatment. The BWS with an exoskeleton, such as the ReoAmbulator gait training robot [11], which almost completely limits the motion of the trunk and pelvis, has the drawback that these robots may limit the synergic movement of the whole body. In the similar way, the BWS with footplate devices, such as G-EO system [12], Gait Master [13], and Haptic Walker [14], shows that these robots control the position and orientation of the foot to implement the gait motion. As for control, the Lokolift of the Lokomat [15] is to provide precise body weight unloading for patients via a passive elastic spring element to take over the main unloading force and an active closed-loop controlled electric drive to generate the exact desired force. But, stroke patients show exaggerated lateral excursions of the pelvis caused by muscular weakness and the BWSs with the exoskeleton usually limit the pelvic motions. To correct these pathological movements, a Pelvic Assist Manipulator (PAM) has been designed by Aoyagi et al. [16] which has five active degrees of freedom to control the pelvic motions. A problem that follows is that the active participation of the patient is key for motor relearning. To encourage these patients for active involvement, Pietrusinski et al. [17] designed a robotic gait rehabilitation (RGR) trainer to correct pelvic obliquity using a force-field controller.

However, the research on the PBWS with the footplate device and pelvic mechanism remains to be performed. Thus, a novel RGT is presented to help with sit-to-stand transfer, active gait training, and balance function assessment in this paper, and the advantages of this design are given as follows: (i) to provide users with bilateral body weight support and meanwhile help with the active control of pelvic obliquity; (ii) to meet the needs of the pelvic motions (pelvic tilt, pelvic rotation, lateral motion and forward-backward motion) passively; (iii) to combine the PBWS and the BE to control the lower limb movements, such as *Hip Flex./Ext.*, *Knee Flex./Ext.*, and *Dorsi. Flex.*

The rest of this paper is organized as follows: In Section 2, the system description of the robot is detailed. The kinematics of the robot is presented in Section 3. Simulation analyses such as workspace, sit-to-stand process, and movement trail analysis are conducted in Section 4. Finally, conclusions and future work are given in Section 5.

## 2. System Description

The RGT focused on the realization of sit-to-stand transfer, active gait training, and balance function assessment for patients. The RGT consists of a bilateral BWS system, bipedal end-effector, screen, control cabinet, and pelvic brace. The BE has two robotic arms under a speed control to meet the needs of the motions of lower limbs. The PBWS has two linear guideways that provides sit-to-stand transfer and mass-offloading. The pelvic brace is to detect the interactive signal and smooth the pelvic motions.

### 2.1. Description of the System

This paper aimed to apply engineering knowledge to solve clinically relevant problems, so the rehabilitation demands of targeted subjects should be figured out. The pelvic motions play an important role in normal gait and body balance [18, 19]; the lateral and vertical motions of the pelvis, pelvic obliquity, and rotation are the key parameters for body stabilization [20]. According to the previous work, the normal range of the pelvic motions during gait is given in [21]. Therefore, the RGT is designed to provide lower limb assistance and pelvic movement assistance.

Figure 1 shows the three-dimensional model of the RGT with a dummy. The robot consists of three main parts: (i) a bipedal end-effector (BE), which is controlled by six servo motors to implement the biped gait trajectory so the BE offers the feature of realistically simulating walking and climbing stairs; (ii) a bilateral body weight support system (PBWS), which is controlled by two servo motors to implement mass-offloading and pelvic obliquity; (iii) a pelvic brace (PB). Screen interaction, physical sensors, and other accessories are involved in the robot. The BE consists of two robotic arms (three DoFs for each arm, driven by three servo motors of Beckhoff Co. Ltd.), to control the position of the foot in the vertical plane and posture of the foot, so that the user can walk on the RGT. The PBWS is mounted on the BE via a height setting; the purpose of the PBWS is to provide the force assistance during the standing/sitting process and body weight support in the vertical direction during walking. The PBWS is designed to realize the control of pelvic obliquity via different heights of both sides of the pelvis. Between the PBWS and the subject, the PB is designed to connect the robot. The PB is mounted at the end of the PBWS and consists of two torque sensors (double flange, 200 Nm), the lateral motion mechanism (realized by two ball splines), the pelvic rotation mechanism (realized by two linear guideways), and four pressure sensors (cylindrical tension/pressure sensor).

The pelvic rotation mechanism and the lateral motion mechanism are equipped with reset springs, and thus, the pelvis of the user will perceive the feedback force when his/her pelvis deviates away from the equilibrium position. Four pressure sensors are installed on the two sides of the user; details on the method of application follow shortly. The data collection, signal processing, and movement control are done on the controller.

### 2.2. Control Algorithm

The control of the RGT is divided into two stages, (i) passive mode, the RGT implements the gait cycle when the subject is not capable of walking (to correct the pathological movements); (ii) active mode, the RGT detects the motion intention of the subject and assists them in finishing the gait cycle (to encourage the patients for active involvement). For the active mode, as shown in Figure 2, the RGT monitors the interaction forces through the two torque sensors and four pressure sensors first and then the controller calculates the resultant force and recognizes the motion intention of the user; finally, the controller outputs the driving velocity of robot joints via the robot kinematics.

During the operation of the RGT, the user applies forces on the two torque sensors and four pressure sensors to maneuver the robot. These interactive signals are sent to the controller to determine the corresponding walking intention and trajectory of the foot. With the user's intention and motion states of the robot, the controller will generate proper motor speeds to assist the user. For the passive mode, the trajectory of the foot is settled. However, the control of the PBWS is based on the interactive signals. As shown in Figure 3, the mass of the user and the interactive signals are system inputs, *F*_*d*_ is the desired support force, *F*_*s*_ is the resultant force in the vertical direction, and the height of pelvis is monitored using the encoder to optimize the output velocity. When the user walks on the robot, the displacement of pelvis (vertical direction) will motivate the two torque sensors and then the system can calculate the error between the desired force and the resultant force; the error *e*_*b*_ and its differentiation ${\dot{e}}_{b}$ are defined as

(1) $$\begin{array}{c} e_{b}=F_{d}-F_{s},\\ {\dot{e}}_{b}={\dot{F}}_{d}-{\dot{F}}_{s}. \end{array}$$

For the time-varying pelvic position, the resultant force is periodic. Hence, the pelvic velocity *v*_*p*_′ is considered to optimize the output velocity. After Kalman filtering, the speed feedback control method (PD controller) is used to eliminate the tracking error. The output velocity *ν*_*m*_ of the RGT can be expressed as

(2) $$\begin{array}{c} \nu_{m}=k_{p}e_{b}+k_{d}{\dot{e}}_{b}+k_{v}v_{p}^{\prime }, \end{array}$$

where *k*_*p*_ and *k*_*p*_ are the PD parameters of the control algorithm and *k*_*v*_ is the gain of velocity. To calculate the output velocity of each motor of the BE, kinematical modeling is required.

## 3. Kinematical Modeling

Figure 4 shows the kinematic model and coordinate system of the RGT, depicting the motion principle of each joint and overall structure of the robot. The BE contains joints 1∼3 and joints 7∼9, the PBWS contains joint 4 and joint 10, and the PB contains joints 5 and 6 and joints 11 and 12. In this paper, the vectorial method is used for kinematic modeling [22].

*o*_0_ *x*_0_ *y*_0_ *z*_0_ is the local coordinate system attached to the robot. *o*_*i*_*x*_*i*_*y*_*i*_*z*_*i*_ is the *i*th joint coordinate system, and *o*_*p*_*x*_*p*_*y*_*p*_*z*_*p*_ is the joint coordinate system attached to the pelvic center. The position and orientation of the pelvic center are defined as $p_{R}={\left[\begin{array}{ccc} x_{p} & y_{p} & z_{p} \end{array}\right]}^{T}$ and $o_{R}={\left[\begin{array}{ccc} \alpha & \beta & \gamma \end{array}\right]}^{T}$. $\nu_{q}={\left[\begin{array}{cccc} {\dot{q}}_{1} & {\dot{q}}_{2} & \ldots & {\dot{q}}_{12} \end{array}\right]}^{T}$ is the joint velocity of the robot, where the joints of PB are passive (blue arrows) and the rest of joints are active (red arrows). ${\left[\begin{array}{cccc} l_{1} & l_{2} & \ldots & l_{12} \end{array}\right]}^{T}$ is the bar length of the robot. According to the analysis and derivation, the velocity of the motor $\nu_{q}={\left[\begin{array}{cccc} {\dot{q}}_{1} & {\dot{q}}_{2} & \ldots & {\dot{q}}_{12} \end{array}\right]}^{T}$ is solved. For the rigid body system with *n* joints, the position of endpoint can be expressed as ^0^**P**_*n*+1_=∑_*i*=0_^*n*^^0^**R**_*i*_**b**_*i*_′, where ^0^**R**_*i*_ is the rotation matrix from the 0th frame to the (*i* − 1)th frame and **b**_*i*_′ is the position vector from the *i*th joint to the (*i* + 1) joint in the *i*th local frame. As shown in Figure 5, the displacement of the right ankle in the sagittal plane can be expressed as

(3) $$\begin{array}{c} a_{yr}=-l_{1}+q_{1}+\cos\;q_{2}l_{2}, \end{array}$$

(4) $$\begin{array}{c} a_{zr}=\sin\;q_{2}l_{2}. \end{array}$$

And, the displacement of the right hip in the sagittal plane can be approximatively expressed as

(5) $$\begin{array}{c} h_{yr}=q_{6}, \end{array}$$

(6) $$\begin{array}{c} h_{zr}=q_{4}. \end{array}$$

Then, the vector from the right ankle to right hip can be expressed as

(7) $$\begin{array}{c} {\vec{l}}_{ahr}={\left[\begin{array}{cc} a_{yr}-h_{yr} & a_{zr}-h_{zr} \end{array}\right]}^{T}. \end{array}$$

Once the length of legs (thigh *l*_*t*_ and shank *l*_*s*_) is obtained, the lower limb joint angles (right hip *θ*_*hr*_, right knee *θ*_*kr*_, and right ankle *θ*_*ar*_) can be expressed as

(8) $$\begin{array}{c} \theta_{hr}=\theta_{t2r}-\theta_{t1r}, \end{array}$$

(9) $$\begin{array}{c} \theta_{kr}=\pi -\cos^{-1}\left(\frac{l_{t}^{2}+l_{s}^{2}-l_{ahr}^{2}}{2l_{t}l_{s}}\right), \end{array}$$

(10) $$\begin{array}{c} \theta_{ar}=q_{3}-q_{2}, \end{array}$$

where *θ*_*t*2*r*_ is the intersection angle between the vector ${\vec{l}}_{ahr}$ and the vertical vector and the *θ*_*t*1*r*_ is the intersection angle between the vector ${\vec{l}}_{ahr}$ and the vector ${\vec{l}}_{t}$. The aforementioned intersection angles can be calculated via the trigonometric function. And, the joint angles of left leg can be obtained in the similar way.

For the pelvic motions, the vertical motion *z*_*p*_ and the pelvic obliquity *β*_*p*_ are controlled by the robot, the pelvic tilt is unrestricted, and the pelvic rotation *γ*_*p*_, lateral motion *x*_*p*_, and forward-backward motion *y*_*p*_ are satisfied passively:

(11) $$\begin{array}{c} x_{p}=q_{5}, \end{array}$$

(12) $$\begin{array}{c} y_{p}=\frac{q_{6}+q_{12}}{2}, \end{array}$$

(13) $$\begin{array}{c} z_{p}=\frac{q_{4}+q_{10}}{2}, \end{array}$$

(14) $$\begin{array}{c} \beta_{p}=\sin^{-1}\left(\frac{q_{4}-q_{10}}{l_{p}}\right), \end{array}$$

(15) $$\begin{array}{c} \gamma_{p}=\sin^{-1}\left(\frac{q_{6}-q_{12}}{l_{p}}\right), \end{array}$$

where *l*_*p*_ is the width of the pelvis.

Now, the next step is to calculate the joint angles via the desired motion trajectory. The magnitude of the vector ${\vec{l}}_{ahr}$ (the joint angle *θ*_*kr*_ is determined) can be expressed as

(16) $$\begin{array}{c} l_{ahr}=\sqrt{l_{t}^{2}+l_{s}^{2}-2l_{t}l_{s}\cos\left(\pi -\theta_{kr}\right)}. \end{array}$$

Then, the 1th joint angle can be expressed as

(17) $$\begin{array}{c} q_{1}=l_{1}+\cos\;q_{2}l_{2}-q_{6}-\sin\left(\theta_{t1r}-\theta_{hr}\right)l_{ahr}, \end{array}$$

where *θ*_*t*1*r*_ is the intersection angle between the vector ${\vec{l}}_{ahr}$ and the vector ${\vec{l}}_{t}$. To solve *q*_1_, *q*_6_ and *q*_2_ are required. The 6th joint angle can be expressed as

(18) $$\begin{array}{c} q_{6}=y_{p}+\frac{\sin\;\gamma_{p}l_{p}}{2}, \end{array}$$

and the 2th joint angle can be expressed as

(19) $$\begin{array}{c} q_{2}=\;\sin^{-1}\left(\frac{q_{4}-h_{t1r}}{l_{2}}\right), \end{array}$$

where *h*_*t*1*r*_=cos(*θ*_*t*1*r*_ − *θ*_*hr*_)*l*_*ahr*_. The 4th joint angle can be obtained from the pelvic motions:

(20) $$\begin{array}{c} q_{4}=z_{p}+\frac{\sin\;\beta_{p}l_{p}}{2}. \end{array}$$

The 3rd joint angle and 5th joint angle can be expressed as

(21) $$\begin{array}{c} q_{3}=\theta_{ar}+q_{2},\\ q_{5}=x_{p}. \end{array}$$

## 4. Simulation Study

The workspace and the force field of the RGT are calculated based on the kinematical modeling and motion trajectories of the lower limbs [23], and control simulation is carried out to analyze the processes of the sit-to-stand (STS) transfer and gait training.  Figure 6 shows the mean motion trajectories of the lower limbs collected from the motion capture system, and these motion trajectories are used to represent the joint motions of the user during normal walking. The simulation results indicate that the RGT can satisfy the demand of the STS transfer and normal walking.

### 4.1. Workspace Analysis

The workspace of the RGT is shown in Figure 7, the green dots represent the reachable points of the pelvic center, Figure 7(a) shows the positional space, and Figure 7(b) shows the orientation space. The workspace is calculated from kinematic modeling (equations (3)∼(15)) and determinate spring stiffness. To satisfy the required range of motion (RoM) of the lower limbs and pelvis, the workspace analysis of the RGT is studied.

The positional workspace was determined by the passive joint variables referring to the BWSS. Combining the kinematic modeling and determinate spring stiffness, the positional workspace is calculated via MATLAB as shown in Figure 7. According to the positional workspace and motion trajectory of the pelvic center, as shown in Figure 8, the RGT can provide the user with sufficient motion space during normal walking. Besides, the orientation workspace is sufficient by comparison between Figures 6 and 7(b).

In the positional workspace, the deformation of the springs will cause the feedback force to guide the pelvis to the equilibrium position. The motivation of the feedback force is to limit the exaggerated irregular motions, and its magnitude can be calculated via the static Jacobian measure [24, 25]. With defined stiffness of springs and kinematics, the force field in the positional workspace is shown in Figure 9. As can be seen from Figure 9, the maximal magnitude of the feedback force is less than 75 N and the minimum magnitude of the feedback force is 0 N, located in the equilibrium position. Furthermore, the feedback force increases with the deviation from the equilibrium position, which is potential for correction of pelvic motions [26].

### 4.2. Control Simulation

The simulation results are shown in Figures 10 and 11. In the simulation process, the parameters of the system are defined first, then the motion trajectories of the lower limbs and kinematics are inputted into MATLAB, and after that, the inverse Jacobian model can be obtained. Furthermore, we can change the parameter sets of the model, such as the length of the thigh, the length of the shank, and range of motions, to control the motion trajectories of the robot. The next step is to define the positional workspace of the ankle and pelvis. The last step is to calculate the angular velocities of the six motors of the BE.

Figure 10(a) shows the result of the simulation of gait training, the green dots represent the reachable points of the ankle, and the black line represents the motion trajectory of the ankle during the gait process.  Figure 10(b) shows the result of the simulation of the STS transfer process, the green dots represent the reachable points of the pelvic center, and the black line represents the motion trajectory of the pelvic center during the STS transfer process. As can be seen from Figure 10, the RGT can cover the motion requirements of the user.  Figure 11 shows the results of the simulation of the joint angles in a gait cycle, and it can be used to optimize the joint space of the robot.

## 5. Conclusions

This paper introduces a novel robot-assisted gait trainer with the PBWS to assist the elderly and the disabled during the STS transfer and gait training. Kinematical modeling, control algorithm, and simulation study were proposed to analyze the usability of the system, and the motion trajectories of the foot and pelvis are planned based on the clinical-relevant data. The preliminary results showed that the gait trainer can provide the pelvis with sufficient workspace with dexterity and adequate space for gait training. The present work demonstrates the potential capability of the novel robot, and a new method is presented to support the body weight without affecting the pelvis motions. The future work is to complete the manufacture of the robot and investigate the effectiveness of rehabilitation.

## Figures and Tables

**Figure 1:** Schematic diagram of the robot-assisted gait trainer.

**Figure 2:** Illustration of the human-machine interaction.

**Figure 3:** Control architecture of the BWSS.

**Figure 4:** Schematic diagram and coordinate system of the RGT.

**Figure 5:** Vector in the sagittal plane.

**Figure 6:** Motion trajectories of the lower limbs in a gait cycle. “R_” denotes the right, and “L_” denotes the left. The blue solid line denotes the mean motion trajectories of the lower limbs.

**Figure 7:** The workspace of the RGT (green dots); the coordinate unit is meter. (a) Positional space. (b) Orientation space.

**Figure 8:** The motion trajectory of the pelvic center during normal walking (black line) and simulative trajectory (dash-dotted line). The coordinate unit is meter.

**Figure 9:** Simulation results of the force field in the positional workspace. The HSV color scale encodes the norm of force vector in the space; yellow indicates areas with a higher force vector.

**Figure 10:** Simulation results of the gait and the STS transfer process. (a) Positional space of the ankle. (b) Positional space for the STS.

**Figure 11:** Simulation results of the joint angles in a gait cycle.

## Data Availability

The simulation results and experimental results data used to support the findings of this study are available from the corresponding author upon request.
